# Cefepime-Induced Neurotoxicity in a 74-Year-Old Woman

**DOI:** 10.7759/cureus.21918

**Published:** 2022-02-04

**Authors:** Samanvaya Sharma, Muzammil Khan, Muhammad Owais, Asim Haider

**Affiliations:** 1 Internal Medicine, Renaissance School of Medicine at Stony Brook University, Stony Brook, USA; 2 Internal Medicine, Stony Brook University Hospital, Stony Brook, USA; 3 Respiratory Medicine, Rush University Medical Center, Chicago, USA; 4 Internal Medicine, BronxCare Health System, New York, USA

**Keywords:** electroencephalogram, cephalosporin, seizures, cefepime, neurotoxicity

## Abstract

Cefepime is a fourth-generation cephalosporin with anti-pseudomonal coverage. It has been known to cause neurotoxicity, especially in critically ill patients and those with renal impairment. This neurotoxicity is poorly characterized and under-recognized. We present a case of cefepime-induced neurotoxicity in a 74-year-old woman being treated for cellulitis and osteomyelitis. Symptoms were gradual in onset and included confusion, verbal perseveration, and myoclonus. EEG findings included generalized periodic discharges (GPD) and generalized rhythmic delta activity with admixed sharps (GRDA + S). Symptoms resolved one to two days after the cessation of cefepime and anti-epileptic therapy with lorazepam, topiramate, and levetiracetam. We follow this with a discussion of available literature and recommend regular therapeutic drug monitoring in the future.

## Introduction

Cefepime is a fourth-generation cephalosporin, a well-known broad-spectrum antibiotic with antipseudomonal coverage and some resistance to beta-lactamases. It was made commercially available in 1994 [1]. Since 1999, it has been known to cause neurotoxicity, a side-effect that is under-recognized and poorly studied. We present here a case of cefepime-induced neurotoxicity (CIN) followed by a discussion of its salient features with the associated literature. It is our hope that our work will contribute to a greater awareness of CIN, ultimately curbing the associated morbidity for patients.

## Case presentation

A 74-year-old woman with a history of peripheral vascular disease, stage 3b chronic kidney disease, type 2 diabetes mellitus, and anxiety presented to the emergency room for urgent management of a foot ulcer and associated cellulitis upon the recommendation of her vascular surgeon in the clinic. She had been complaining of severe pain at the site worsening over the course of one week. The review of systems was otherwise negative. Vital signs were within normal limits. On examination, her wound revealed an exposed tendon with a malodorous necrotic soft tissue base. The laboratory findings are given in Table 1. 

**Table 1:** Laboratory findings

Laboratory parameter	Laboratory value
Erythrocyte sedimentation rate	45 mm/hr (Range: 0 to 29 mm/hr)
C-reactive protein	0.9 mg/dl (Range < 0.3 mg/dl)
Blood urea nitrogen	47 mg/dl (range: 6-24 mg/dl)
Creatinine, Serum	1.3 mg/dl (Range: 0.7-1.5 mg/dl)
White blood cells	5.1 k/ul (range: 4.8-10.8 k/ul)

A foot radiograph and CT ruled out fracture and gas gangrene. A foot MRI identified multiple foci suggestive of osteomyelitis. The patient was started on empiric cefepime 2g Q12H and vancomycin for cellulitis and osteomyelitis, methocarbamol, gabapentin, oxycodone, and pro re nata (PRN) morphine for analgesia, fluids for prerenal acute-on-chronic kidney injury, and admitted for further management as per podiatry and vascular surgery recommendations. Wound culture was positive for *Klebsiella oxytoca* (sensitive to cefepime), *Serratia liquefaciens* (sensitive to cefepime), and alpha-hemolytic Streptococci (Viridans group). Blood cultures were positive for coagulase-negative staphylococci. An antibiotic regimen was continued as initiated.

On day two of the hospital course, the patient was found to be confused and delirious. A finger stick blood glucose test was 41 mg/dL, prompting the administration of dextrose 50 in water leading to improvement in mentation. Her basal insulin regimen was accordingly adjusted. A few hours later, however, the patient was found to be confused again, repeatedly saying her first name in response to all questions and unable to follow any instructions. This time, her fingerstick glucose test was normal. A non-contrast head CT and a CT angiogram of the head and neck ruled out any acute cerebrovascular pathology (Figure 1).

**Figure 1:** CT scan of the head showing no acute pathology

These findings were confirmed with an MRI. The patient then went on to develop rigidity in all four extremities - more severe on the right - with mimicking and automatisms, followed by a rapid return to baseline in two to three minutes. She was started on continuous EEG with video monitoring, identifying generalized background slowing, and rare, very brief runs of generalized rhythmic delta activity (GRDA) over the course of 24 hours. However, given the high risk of seizure with old infarcts and ongoing infection, she was started on levetiracetam 500 mg Q12H for seizure prophylaxis. The leading etiology of the patient’s altered mental status at this time was suspected to be polypharmacy. Her pain regimen was accordingly adjusted, lowering the frequency of methocarbamol, gabapentin, and PRN morphine, and discontinuing oxycodone.

The next few days in the hospital course were marked by mild confusion - the patient was disoriented to time and would often repeat her first name unprompted - and anxiety, which improved with 2 mg of diazepam (home dose) each day. Mental status was otherwise stable. She underwent management of her wound as directed by podiatry and vascular surgery.

On day eight of the hospital course, the patient was not answering any questions and had fluctuating attention. She was unable to follow commands and often stared blankly at interviewers. She was notably pale and was breathing rapidly. She was also noted to have right upper extremity myoclonus. Vitals were significant for tachypnea to 26 breaths/min but otherwise normal. Laboratory studies had no significant acute changes. The patient was again placed on continuous EEG with video monitoring, revealing continuous bursts of high voltage rhythmic 1-2 Hz generalized periodic discharges (GPD). The patient was given lorazepam 2 mg, which broke the EEG pattern for approximately 10 hours, becoming frequent generalized rhythmic delta activity with admixed sharps (GRDA + S). Generalized background slowing was seen again, consistent with the previous EEG. Additionally, the patient’s levetiracetam was raised to 750 mg Q12H and she was also started on topiramate 100 mg QD. A clinical diagnosis of cefepime toxicity was made, and she was switched to ceftazidime 2g Q24H. Additionally, methocarbamol and PRN morphine were discontinued, leaving only reduced-dose gabapentin for analgesia, which was a successful regimen. Delirium precautions were undertaken.

On day nine of the hospital course, the patient’s mental status began to improve. Early in the day, EEG revealed occasional (<9% of the record), brief bursts of GRDA + S, and occasional GPDs with sharp wave morphology at 1 Hz. As the day progressed, there was a significant improvement, and the only significant finding was generalized background slowing consistent with baseline. By day 10, she was conversant and comfortable during the examination. She was continued on ceftazidime, levetiracetam, and topiramate and had no further episodes of altered mental status during the hospital course.

## Discussion

CIN is a generally under-recognized condition, leading to a paucity of data. Studies attempting to identify an incidence rate have ranged significantly in their results. Retrospective studies of febrile neutropenic patients with mildly impaired renal function and ICU patients showed CIN incidence rates of 20% and 15%, respectively [2,3]. In contrast, retrospective studies attempting to find a CIN incidence rate in healthy patients have reported numbers from 6%, 11%, and 23.2% depending on how strictly they define CIN and how broad a section of patients they measure cefepime trough levels in [4-6].

In a systematic review of literature spanning from January 1980 (roughly corresponding to the earliest use of cefepime) to February 2016, Payne et al. reviewed 37 qualifying publications, representing 135 patient cases of CIN [1]. All patients reportedly had altered mental status, most commonly experiencing reduced consciousness (47%), confusion (42%), and myoclonus (42%). Changes in mental status usually appear before myoclonus and seizures. All patients who had EEG data had EEG abnormalities. Symptoms were often delayed with a median onset of four days (interquartile range of two to six days). Treatment usually involved cessation or dose- reduction of cefepime (85% of cases), and sometimes also included antiepileptic drugs - mostly a benzodiazepine- (36% of cases) and, rarely, hemodialysis (8% of cases) [1]. Clinical improvement was observed in a median of two days after intervention (interquartile range of one to three days). Of the patients, 80% had renal dysfunction and 81% with a reported location were ICU patients [1].

These findings are generally reflected in our patient with a few variations. Our patient was confused and verbally perseverating on her name on day two of her cefepime course. The cause of her symptoms was initially suspected to be hypoglycemia, and then polypharmacy, which were both managed accordingly. An EEG revealed background slowing and rare, very brief runs of GRDA. Given the high risk of seizure with her old infarcts and ongoing infection, she was started on levetiracetam on the same day. Cefepime toxicity was not highly suspected, likely due to its limited recognition. The next few days were marked with continued confusion and verbal perseveration on occasion but relatively well-controlled symptoms. Her symptoms exacerbated significantly on day eight of her hospital course. It is impossible to say with certainty whether her altered mental status until this point was entirely or only partially due to cefepime toxicity. Therefore, the onset of symptoms was anywhere between day two and day eight, a range that is likely influenced by her seizure prophylaxis with levetiracetam. Regardless, consistent with the findings reported by Payne et al., she clearly had a period of confusion before developing myoclonus and other motor symptoms [1]. The diagnosis of CIN followed by the cessation of cefepime, one-dose lorazepam, and continued maintenance on levetiracetam and topiramate led to a rapid resolution of symptoms within one to two days, as is reportedly typical. Lastly, our patient had stage 3b chronic kidney disease, so for her to be at significant risk for developing CIN would also be consistent with the findings of Payne et al. [1].

Boschung et al. concluded that in the patients with risk factors for developing the CIN, cefepime trough levels should be routinely measured and maintained to be < 7.5 mg/L [6]. The clinical symptoms of CIN include headache (<1%), aphasia (<1%) [7], confusion (<1%), encephalopathy (<1%), seizure (<1%) [8], hallucination (<1%) [2], myoclonus (<1%) [9], status epilepticus (<1%) [10], stupor (<1%) [11], and coma (<1%) [12]. These adverse effects can occur even with the appropriate dosing and usually resolve once the drug is interrupted; however, some patients may require additional interventions (e.g. antiepileptic therapy or hemodialysis) [1].

## Conclusions

We conclude by reiterating that CIN is under-recognized. When cefepime is administered to patients with renal impairment, CIN must be considered on the differential if patients develop altered mental status, myoclonus, convulsive seizures, or nonconvulsive status epilepticus. EEG findings are abnormal in every known case of CIN, and therefore clinicians should not hesitate in placing these patients on EEG monitoring upon any mental status alterations. We also recommend routine monitoring of cefepime trough levels in patients on cefepime - particularly patients with renal impairment - and we emphasize the need for prospective studies in this regard to identify a clear threshold.
